# Efficacy of Pretreatment with *Lycium barbarum* Polysaccharide in Various Doses in Influencing Splenic Immunity and Prognosis of Sepsis in Rats

**DOI:** 10.1155/2022/9508603

**Published:** 2022-10-04

**Authors:** Huan Ding, Ping Yang, Xue-hong Zhang, Yu-Jie Ma

**Affiliations:** ^1^Department of Critical Care Unit, General Hospital of Ningxia Medical University, Niangxia 750004, China; ^2^Department of Emergency, General Hospital of Ningxia Medical University, Niangxia 750004, China; ^3^Department of Pediatrics, Shenzhen Union Hospital, Huazhong University of Science and Technology, Gaung Zhou 518052, China

## Abstract

**Objective:**

Sepsis, showing high mortality, is a lethal dysfunction of organs caused by an infection-induced disorder in the host response. It has complicated pathogenesis, which has not yet been elucidated completely. Recently, the principal factors causing pathogenesis and even death in sepsis patients are imbalance in inflammatory response and immunosuppression occurring when the host is challenged by infection. Previous studies found that *Lycium barbarum* polysaccharide (LBP) worked well in enhancing immunity. This study aims at exploring the efficacy of pretreatment with LPB in regulating splenic immunity during the pathogenesis of sepsis induced by cecum ligation perforation (CLP) in rats.

**Methods:**

This research established the cecum ligation perforation rat model. Using immunohistochemistry and flow cytometry, the effects of *Lycium barbarum* polysaccharide in various doses in influencing splenic immunity and prognosis of sepsis induced by cecum ligation perforation in rats were examined.

**Results:**

This study showed that LBP lowered the 72-hour mortality of sepsis rats induced by CLP, relieved systemic inflammation, improved the ratio of T-cell subgroups positive in CD3+, CD4+, or CD8+ and expression of HLA-DR protein, and repaired damage to splenic tissue, implying its efficacy in enhancing the immunity of sepsis rats induced by CLP.

**Conclusions:**

LBP may ameliorate clinical symptoms of rats with cecum ligation perforation, improve cellular immunity in the spleen, and treat sepsis so as to provide a theoretical basis for the pathogenesis and development of sepsis as well as its diagnosis and treatment, and offer scientific proof for the development and utilization of LBP applied to critical diseases.

## 1. Introduction

Sepsis, showing high mortality, is a lethal dysfunction of organs caused by an infection-induced disorder in the host response [1]. It has complicated pathogenesis, which has not yet been elucidated completely. Recently, the principal factors causing pathogenesis and even death in sepsis patients are imbalance in inflammatory response and immunosuppression occurring when the host is challenged by infection. These inappropriate reactions induce depletion of immune cells such as T lymphocytes and alteration of their functions, thereby resulting in dysfunction of organs [2, 3].

During the past several decades, therapeutic strategies for sepsis have been centered on control of infection, liquid resuscitation, mechanical ventilation, organ protection, and nutritional support. Despite the great progression achieved recently in the improvement of immune function in sepsis patients, their mortality remains at a high level [4]. The reason lies in that most of the patients can survive severe systemic inflammation, owing to the improvement in supportive treatment, and enter the phase of immunosuppression seeming more sophisticated. Under the effect of immunosuppression, secondary infection occurs more often in sepsis patients who may die because of uncontrollable infection [5]. Immune-modulating therapy, therefore, has become the most important approach in the treatment of sepsis, and the focus of research is on how to inhibit nonspecific inflammatory reactions in sepsis patients, improve the function of their immune organs, and avoid injuries of tissues and cells.

*Lycium barbarum* L, one of the specific traditional Chinese herbs in Ningxia belonging to Solanaceae Lycium, is the mature dried fruit of Ningxia *Lycium barbarum* with homology in both food and medicine. Its main ingredients include *Lycium barbarum* polysaccharide (LBP), lycium pigment, glycine betaine, atropine, and celestial amines, among which LBP is the main ingredient exerting the pharmacological actions of this drug. LBP, a water-soluble polysaccharide, is capable of fighting against oxidative stress [6], lowering blood glucose and lipids [7], delaying senility [8], protecting nerves [9], treating tumors [10], protecting the liver [11], and improving and regulating immunity [12,13]. Celestial amines have been adopted as the adjuvant drugs applied to diseases correlated to immunosuppression, such as cancers. The efficacy of LBP to improve the proliferation of T cells and ameliorate immunity has been confirmed by a great number of animal experiments [14]. LBP research studies at present, however, are focusing on chronic diseases such as diabetes and on acute diseases centered on injuries of the organs including the retina [15], heart/cerebral ischemia, and reperfusion [16,17], and hepatic oxidative stress [11], while studies seem insufficient on LBP-regulated immunity in sepsis patients. T lymphocytes may reflect systemic immunity [18,19], while HLA-DR is the important marker influencing prognosis of sepsis [20]. This research is based on these arguments and aims to discuss the efficacy of pretreatment with LBP in influencing splenic immunity and prognosis in rats with sepsis induced by cecum ligation perforation (CLP).

## 2. Material and Method

### 2.1. Chemicals

Chemical reagents and antibodies used in this research included: rat TNF-alpha Platinum ELISA (eBioscience, USA), rat IL-10 Platinum ELISA (eBioscience, USA), anti-rat CD3 PE (eBioscience, USA), anti-rat CD4 APC (eBioscience, USA), anti-rat CD8 FITC (eBioscience, USA), rabbit anti-mouse HLA-DR monoclonal antibody (Abcam, UK), and LBP in analytical grade (Bar Ruiyuan, Yinchuan, China). Take 15 g of *Lycium barbarum* polysaccharide powder with a purity of 53% and dissolve it in 30 ml of 0.9% sodium chloride injection to prepare an LBP solution with a concentration of 50%. Different doses of 200 mg/kg, 400 mg/kg, and 800 mg/kg (i.e., 0.2 ml/250 g, 0.4 ml/250 g, and 0.8 ml/250 g) of LBP solution were given to the rats by gavage, respectively, according to the body weight of the rats, and LBP was increased according to the body weight of the rats.

### 2.2. Experimental Animals and Experimental Groups

100 healthy male clean Sprague Dawley (SD) rats (aged 8 weeks and weighing 250 ± 20 g) were provided by our university. The number of animal qualification certificate is SYXK (Ning) 2015-0016. All animals were bred under the same climate, ventilation condition, temperature, and humidity conditions indoors with 12 h day and night alteration. All animals were provided with the same diet including one week of adaptive feeding, before randomization into five groups (in Table 1), including (1) the Sham, (2) cecum ligation perforation (CLP), (3) CLP rats treated with 200 mg/kg LBP (LPB1), (4) CLP rats treated with 400 mg/kg LBP (LPB2), and (5) CLP treated with 800 mg/kg LBP (LPB3). A 2-week lavage was performed, followed by replication of sepsis induced by CLP, and division further for each group into 3 subgroups (6 h, 12 h, and 18 h) based on modeling time (Table 1). All experiment protocols were authorized by the Laboratory Animal Management Committee of Ningxia Medical University (2019-208), consistent with guidelines on animal ethics issued by the National Institute of Health.

### 2.3. Treatment with Drugs

Lavage with various doses (200 mg/kg/day, 400 mg/kg/day, and 800 mg/kg/day) of LBP solution was performed for animals in LBP pretreatment groups. 2 weeks after LBP pretreatment, a sepsis model induced by CLP was established. Animals in Sham and CLP were treated with normal saline in the same volume.

### 2.4. Establishment of the CLP Rat Model

An animal model was established based on methods described in the literature 2 weeks after lavage with LBP, with procedures as follows [21]. The animals were abstained from food (but not from water) for 12 hours before the establishment of models. The rat was anesthetized through intraperitoneal injection with 1% pentobarbital sodium (40 mg/kg per rat), and the operative region of its abdomen was disinfected. A midline incision was made in the lower abdomen, and a 3-0 sterile suture was used to ligate the cecum at 2.5 cm off the cecum end (far end of the ileocecal valve). Then three perforations through the cecum were made with a 22G needle, with an interval of 1 cm between every two perforations, to yield 6 fistulas, through which a little stool was squeezed out. Then closure was performed on the peritoneum, abdominal muscles, and skin, layer by layer. Ringer's solution was injected hypodermically at the neck with a dose of 50 ml/kg as a compensation for intraoperative liquid loss and as an antishock treatment. The rats were kept individually with one animal in each cage and their activities were observed. Except for ligation or perforation of the cecum, which was omitted, incision and closure as well as all other procedures in the Sham Group were identical to those in the CLP Groups. After the operation, the rats were allowed ad libitum to food and water.

Before euthanasia, the clinical score of rats was evaluated at various time points, using the method described by Weber et al. [22] as follows: (a) appearance: normal (0), lack of licking (1), piloerection (2), hunch (3), eyes half open or closed (4); (b) changes in behaviors at rest: normal (0), minor change (1), solitary (2), dysphoria (3); (c) changes in behaviors under exterior stimulation: prompt response (0), response (1), lags in response (2), no response (3); (d) clinical signs: normal respiratory rate (0), minor changes (1), decrease of respiratory rate while manifesting abdominal respiration (2), significant abdominal respiration and cyanosis (3); (e) presence or absence of dehydration: normal (0), dehydrated (5). A higher score corresponds to a worse status of rats. The rats were sacrificed in a closed container by CO_2_ (15 L/min, the volume of the euthanasia chamber is 60 × 50 × 50 cm) and verified death by breathing and pupil (end observation in 30 minutes).

### 2.5. Collection and Preparation of Samples

Blood collection: 6 rats were taken from each group respectively at hours 6, 12, and 18 after CLP and underwent cardiac puncture (1% pentobarbital sodium, 40 mg/kg per rat before puncture) to take a blood sample with the serum separated. 2 ml of whole blood was put in a tube containing no EDTA, kept standing for 2 hours under room temperature, and centrifuged at 700 g/min for 15 minutes to separate serum, which was kept in a −80°C refrigerator until analysis on levels of TNF-*α* and IL-10. Additional 3 ml of whole blood was sampled and put into an EDTA tube, kept standing for 30 minutes at room temperature, and analyzed further with flow cytometry.

Tissue collection: the spleen was taken out from the rat after blood sampling and kept in 10% neutral buffered formalin to be fixed for histopathological analysis.

### 2.6. Clinical Score Assessment

Before the rats were executed, Weber's [22] and other methods were used to evaluate the clinical scores of rats at different time points specifically as follows: (a) appearance: normal (0), lack of combing (1), hair (2), stoop (3), half-open eyes (4); (b) resting state behavior changes: normal (0), slight changes (1), isolation (2), restlessness (3); (c) external stimulus behavior changes: sensitive response (0), reaction (1), slow response (2), no response (3); (d) clinical signs: normal respiratory rate (0), slight change (1), decreased respiratory times and abdominal breathing (2), significant abdominal breathing and cyanosis (3); (e) whether dehydration: normal (0), dehydration (5). The higher the score, the worse the condition of the rats.

### 2.7. Sample Collection and Preparation

Blood collection: six rats were taken from each group at 6, 12, and 18 hours after CLP. Blood samples were collected by heart puncture and serum was separated. 2 ml of whole blood was collected in the blood vessels without EDTA. Serum was collected at room temperature for 2 hours, centrifuged at 700 g/min for 15 minutes, and stored in a −80°C refrigerator for reserve until the levels of TNF-alpha and IL-10 were analyzed. In addition, 3 ml whole blood was collected and placed at room temperature for 30 minutes. Flow cytometry was used for further detection.

Tissue collection: after blood collection, the spleen of rats was further removed and fixed in 10% neutral formalin solution for histopathological analysis.

### 2.8. Enzyme-Linked Immunoassays (ELISAs) of Inflammatory Factors

100 *μ*l of test serum was taken and analyzed for the expression of its inflammatory factors TNF-*α* and IL-10 through an enzyme-linked immunosorbent assay (ELISA).

### 2.9. Detection of Leukocyte Count, Neutrophil Count, and Lymphocyte Count

0.5 ml of anticoagulated peripheral blood was delivered to the Laboratory Department of General Hospital of Ningxia Medical University for testing white blood cell (WBC) count, neutrophil count (NEU), and lymphocyte (LYM) count.

### 2.10. Measurement of Splenic Index

The whole spleen was taken, with water and blood absorbed with filter paper, and weighed. The influence on the splenic index of rats in GLP groups by LBP was described, by calculating the body mass of the spleen based on body weight.

### 2.11. Detection of Ratio of CD3+, CD4+, and CD8+ T Cells in Spleen

Part of the spleen tissue was taken and cut repeatedly with scissors into a paste. Splenic cells were sieved through 200-mesh cell sieves and centrifuged at 700 g/min for 10 minutes. Then, the supernatant was taken and added with a lymphocyte separation medium, with splenic cells separated through a Ficoll-Paque density gradient centrifuge. Flow cytometry was used to detect the ratio of CD3+, CD4+, and CD8+ T cells.

### 2.12. HE Staining of Spleen

Part of the spleen was taken and put into 10% neutral buffered formalin to be fixed for histopathological analysis. The sample was embedded into paraffin and sliced into 5*μ*m-thick sections, followed by HE stains and observation of spleen injuries.

### 2.13. Immunohistochemistry (IHC)

Paraffin sections for rat spleen were prepared, and the expression and location of HLA-DR protein in the spleen of rats in each group were detected with IHC staining. DP Ctroller 3.1.1.267 Image Acquisition System was used for light-field photography. Factors influencing light intensity were changed to manual adjustment and fixed, and three sections were chosen for each rat in each group. White balance was used for every section. The “hot region” of protein expression was selected under a low power lens, and in the region, five nonredundant high power fields were selected for photography (200×). The images were analyzed with Image Pro Plus 6.0, a full-automatic analyzing system, and HLA-DR protein staining in splenic tissue was calculated.

### 2.14. Statistical Analysis

Statistical analysis: SPSS 23.0 Software was used for the analysis. Measurement data, expressed in mean ± standard deviation (*X* ± *S*), underwent a normality test and a homogeneity test of variance. LSD was used for intragroup comparison or intergroup pairwise comparison, and one-way analysis of variance was used for multigroup comparison if data is in normality with homogeneity in variance. If not in normality without homogeneity in variance, the data underwent a nonparametric test of rank transformation. The *χ*^2^ test was used for counting data. *P* < 0.05 was considered as the statistically significant difference. All statistical tests were two-sided.

## 3. Results

### 3.1. Effects of *Lycium barbarum* Polysaccharide on General Conditions and Clinical Scores of LP Rats at Different Time Points

Clinical manifestations in various degrees were observed in CLP Group and LBP Groups, including mental malaise, piloerection, hair humidity, increased bloody excretion around the eye and mouth, decreased activities, lags in response, decreased respiratory numbers, increased abdominal respiration, cyanosis at extremities, and dehydration. An increase of bloody or purulent exudates in the peritoneal cavity was revealed by abdominal laparotomy, together with turgidity and necrosis of ligated cecum and aggravated adhesion, showing a gradual worsening along with prolongation of modeling. There was no significant change in clinical scores at each time point in the Sham group (*P* > 0.05). Compared with 6 hours, the CLP group and LBP group had higher clinical scores at 12 hours and 18 hours (*P* < 0.01), and the most significant increase at 18 hours (*P* < 0.01). Compared with the Sham group, the CLP group had higher clinical scores (*P* < 0.01) and lower clinical scores than the LBP group (*P* < 0.01), but still, there was no significant difference between the CLP group and the CLP group (*P* < 0.01). The clinical scores of the LBP 2 and LBP 3 groups were lower than those of the Sham group (*P* < 0.01), and the lowest was in the LBP 3 group (*P* < 0.05). (Table 2, Figure 1).

### 3.2. Effect of *Lycium barbarum* Polysaccharide on Serum Inflammatory Factor in LP Rats at Different Time Points

There was no significant change in TNF-a and IL-10 at each time point in the Sham group (*P* > 0.05). Compared with 6 hours, TNF-a and IL-10 in the CLP group and LBP group increased at 12 hours (*P* < 0.01). Compared with 12 hours, TNF-a and IL-10 in the CLP group and LBP group decreased at 18 hours (*P* < 0.01), while IL-10 increased at 18 hours (*P* < 0.01). Compared with the Sham group, TNF-a and IL-10 in the CLP group increased (*P* < 0.01), and CLP <0.01, respectively. Compared with the LBP group, TNF-a in the LBP group decreased (*P* < 0.01), but was still higher than that in the Sham group (*P* < 0.01). Compared with the LBP group, TNF-a in the LBP group and LBP 3 group decreased (*P* < 0.01), IL-10 increased (*P* < 0.01), TNF-a in the LBP group decreased most significantly (*P* < 0.01), and IL-10 increased most significantly (*P* < 0.01) (Figures 2(a)–2(c)).

### 3.3. Effects of *Lycium barbarum* Polysaccharide on LYM in Peripheral Blood of CLP Rats at Different Time Points

There was no significant change in LYM at each time point in the Sham group (*P* > 0.05). Compared with 6 hours, LYM in the CLP group and LBP group decreased at 12 hours (*P* < 0.01), LYM in the CLP group and LBP group decreased at 18 hours (*P* < 0.01), LYM in the CLP group decreased at 18 hours (*P* < 0.01), LYM in the CLP group increased at all time points compared with the CLP group (*P* < 0.01), and the LBP group increased at all time points (*P* < 0.01), compared with the LBP group and LBP group at 12 hours (*P* < 0.01). LYM was increased in the LBP3 group (*P* < 0.01), especially in the LBP3 group (*P* < 0.01).. (Figure 2(d)).

### 3.4. Effects of *Lycium barbarum* Polysaccharide on Splenic Histopathology and Splenic Index of LP Rats at Different Time Points

The histological structure of the spleen in the Sham group was also clear, and the demarcation between red and white pulps was clear. There were a lot of lymphoid nodules (splenic corpuscles) in the white pulp, and there was no significant difference at different time points. In the CLP group, red pulp was congested with edema, splenic sinus was dilated, red pulp and white pulp boundary were blurred, white pulp area was reduced, neutrophil infiltration, macrophage proliferation, lymphocyte nucleus condensation, and fragmentation into multiple apoptotic corpuscles were observed, and the most serious injury occurred in 18 hours. In group B, red pulp congestion was alleviated, the red pulp and white pulp boundary was clear, the white pulp area was enlarged, neutrophil infiltration, macrophage proliferation, lymphocyte nuclear pyknosis and fragmentation were reduced, pathological damage was alleviated compared with the CLP group, and the spleen tissue structure in group LBP3 was best repaired. (Figure 3(a)).

There was no significant change in the spleen index at each time point in the Sham group (*P* > 0.05). Compared with 6 hours, the spleen index of the CLP group and LBP group decreased significantly at 12 and 18 hours (*P* < 0.01), and the spleen index of the CLP group decreased significantly at 18 hours (*P* < 0.01). Compared with the Sham group, the spleen index of the CLP group decreased significantly (*P* < 0.01), and the spleen index of the LBP group increased significantly (*P* < 0.01), compared with that of the CLP group, and the spleen index of the LBP group increased significantly (*P* < 0.01). Compared with the LBP2 and LBP3 groups, the spleen index in the BP1 group increased (*P* < 0.05), and that in the LBP3 group increased most significantly (*P* < 0.05). (Figure 3(b)).

### 3.5. Effects of *Lycium barbarum* Polysaccharide on the Percentage of CD3+, CD4+, and CD8+ T Cells in CPL Rats at Different Time Points

CD3+, CD4+, and CD8+ T cells in the Sham group had no significant changes at each time point (*P* > 0.05). Compared with 6 hours, CD3+, CD4+, and CD8+ T cells in the CLP group and LBP group decreased at 12 h, 18 h (*P* < 0.01), and the most significant decrease at 18 h (*P* < 0.01). Compared with the Sham group, CD3+, CD4+, and CD8+T cells in the CLP group decreased significantly (*P* < 0.01), and compared with the CLP group, the C+, CD8+ T cells in the LBP group decreased significantly (*P* < 0.01). Compared with the LBP1 group, CD3+ (Figure 4), CD4+ (Figure 5), and CD8+ (Figure 6), T cells in the LBP2 and LBP3 groups increased significantly (*P* < 0.05), and those in the LBP3 group increased most significantly (*P* < 0.05). (Figures 4–6).

### 3.6. Effect of *Lycium barbarum* Polysaccharide on HLA-DR Expression in Spleen of LP Rats at Different Time Points

The expression of HLA-DR in the spleen of rats at different time points was semiquantitatively evaluated as negative (−), weak positive (+), positive (++), and strong positive (+++), and membrane binding was evaluated by positive results.

The HLA-DR protein is normally localized in splenic macrophages and B lymphocytes and is mainly expressed in cell membranes. The expression of HLA-DR in the Sham group was positive, showing brown-yellow staining. The brown-yellow region was larger, and the expression intensity was strongly positive (+++), but there was no significant difference between the time points. The brown-yellow staining area of HLA-DR in the CLP group was significantly reduced, the expression intensity was weakened (++), and the brown-yellow staining area of HLA-DR in the LBP group was negative (−) at 18 hours. Compared with the LBP1 group and the LBP2 group, the brown-yellow staining area in the LBP3 group was stronger (+++). There were significant differences in the area of positive staining areas among the five groups (*P* < 0.05) (Figure 7(a)). IOD values of HLA-DR expression in spleen tissues showed that compared with the Sham group, the CLP group decreased significantly (*P* < 0.01) and decreased most significantly at 18 h, while the LBP group increased significantly (*P* < 0.01) and the LBP3 group increased most significantly (*P* < 0.01) (Figure 7(b)).

## 4. Discussion

Cecal ligation and perforation are the gold standards for establishing a sepsis model [21]. In this study, a sepsis rat model was established by cecal ligation and perforation. Two to six hours after the establishment of the CLP model, rats showed shortness of breath, mental fatigue, restlessness, erect hair, and so on. After execution, a small amount of blood exudation was found in the abdominal cavity, and the cecum was swollen at the end of ligation. At 6 to 12 hours, rats showed hypokinesia, lethargy, abdominal distention, chills, increased corner secretion, and disordered hair; after execution, blood exudation in the abdominal cavity increased, the cecum swelling and blackening, adhesion, jejunal tube flatulence, and other manifestations. At 12 to 18 hours, mental depression, body curling, cyanosis at the extremities, corners of the eyes and masks appear bloody secretions; after execution can see abdominal abscess exudation, small intestinal congestion, edema, adhesion, cecum swelling and necrosis and aggravation of the ligation end, stench and other manifestations. In addition, the clinical scores of *Lycium barbarum* polysaccharide pretreated rats were more relieved than those of the CLP group, and the clinical scores of the LBP3 group were lower than those of the CLP group. It is suggested that *Lycium barbarum* polysaccharide can improve the general condition of sepsis rats in a dose-dependent manner.

Inflammatory response is the most principal feature of sepsis, and the initiating factor in its pathogenesis. After the invasion of pathogens into the body, it activates the innate immune system including monocytes, macrophages, and neutrophils, and helps release a great deal of proinflammatory factors such as TNF-*α* and high mobility group box-1 protein (HMGB1), resulting in prolonged excessive inflammation [23, 24]. Meanwhile, the increase in the release of cytokines, including IL-10 and TGF-*β,* activates compensatory anti-inflammatory responses to maintain homeostasis in the internal environment [23]. Our results showed that neutrophils and the inflammatory factors TNF-*α* and IL-10 all rose in the CLP and LBP groups, indicating the presence of excessive systemic inflammatory response. Along with the development of sepsis, the macrophages are inactivated with a reduction of antigen presentation and release of proinflammatory factors in contrast to an increase of anti-inflammatory factors, thereby resulting in immunosuppression. Results of this research showed that TNF-*α* and neutrophils decreased gradually in the CLP and LBP groups in contrast to a persistent increase of IL-10, suggesting that the body was dominated gradually by anti-inflammatory reactions and sepsis entered the status of immunosuppression. Through pretreating sepsis rats with LBP in various doses, we observed decreased release of neutrophils and TNF-*α* in LBP groups in contrast to increased release of IL-10 with more obvious findings in LBP3, suggesting LBP might decrease the excessive inflammatory response in sepsis rats in a dose-dependent manner. Wu et al. [25] found that LBP might reduce the level of TNF-*α* in rats with hepatic injury induced by carbon tetrachloride (CCL4), improve the level of IL-10, and alleviate inflammatory reactions. In macrophage damage in rats induced by lipopolysaccharide (LPS), LBP decreased inflammatory reactions through inhibiting activity of the TLR4/NF-*κ*B pathway and downregulating the expression of inflammatory factors including NO, TNF-*α,* and IL-6 [26]. The capability of LBP to reduce systemic inflammation, as confirmed by these research studies, seems consistent with findings in our research.

Sepsis influences, directly and indirectly, the life span, quantity of all immune cells, and their functions. More and more evidence confirms that immunosuppression plays a central role in inhibiting the development of sepsis. A great loss of immune cells, as confirmed by researchers, exists in sepsis and manifests as a depletion of lymphocytes. Results of this research showed the decrease of lymphocyte count in the CLP and LBP groups, with the most obvious findings at hour 18, suggesting the presence of immunosuppression following a great loss of lymphocytes in CLP sepsis rats along with the prolongation of the disease. After pretreatment with LBP in various doses for CLP rats, an increase of lymphocytes was observed in all groups, with the best outcome in LBP3, implying the capability of LBP to increase the level of lymphocytes of CLP rats and ameliorate their immunity in a dose-dependent manner. T lymphocyte is the important component maintaining homeostasis in systemic immunity, and its apoptosis in great quantity plays an important role in the occurrence of systemic immunosuppression [19]. Our research data showed that the percentage of CD3+, CD4+, and CD8+ T lymphocytes decreased in both the CLP and LBP groups, with a persistent decreasing tendency along with prolongation of time after modeling and the most obvious observation observed at hour 18, suggesting the presence of systemic immunosuppression following a great loss of T lymphocytes in the spleen of CLP rats along with prolongation of the disease. Significant elevation of percentages of CD3+, CD4+, and CD8+ T lymphocytes was noticed in the spleen of LBP groups, with the most obvious rise in LBP3, suggesting the capability of LBP to improve the ratio of T lymphocytes in the spleen of CLP rats and ameliorate splenic immunity in a dose-dependent manner. In the model of tumor-bearing rats induced by doxorubicin, LBP increased peripheral lymphocyte count, recovered cytotoxicity of natural killing cells, and achieved its efficacy in regulating immunity [27], seeming consistent with observations in our research.

As the largest human peripheral immune organ consisting of red pulp and white pulp, the spleen offers an environment for mature T cells to achieve a specific immune response. The splenic white pulp can be divided into the peripheral lymphatic sheath (PLS) and splenic corpuscle (SC, also called lymphoid nodule). The peri-splenic arterial lymphatic sheath comprises an interlaced process between a great number of T cells and a small number of macrophages, while the splenic corpuscle consists of lots of B cells. Observations under the light microscope (Figure 5) showed hyperemia and edema of spleens in the CLP group with enlarged splenic sinus and observable infiltration of neutrocytes in the spleen, where karyopyknosis of lymphocytes was seen followed by fragmentation into lots of apoptotic bodies, with the most severe impairment at hour 18. Given the reduction of the splenic index in CLP rats with more obvious findings at hour 18, the splenic injury seemed probable in sepsis rats induced by CLP, which kept worsening with time and eventually resulted in a decrease in immunity. After treatment with LBP in various doses, CLP rats showed neutrophil infiltration and a decrease in both karyopyknotic and fragmentation of lymphocytes in the spleen, with decreased pathological injuries in comparison with the CLP group, showing the best repair of splenic tissue in the LBP3 group. Considering the increase of splenic indexes in all groups with more obvious findings in the LBP3 group, it could be concluded that pretreatment with LBP might increase splenic indexes of CLP rats and ameliorate the impairment of splenic structure in a dose-dependent manner. Tang et al. [28] found that LBP might decrease splenic index in aged rats, delay atrophy of their spleen, prevent a decrease in immunity, improve proliferation of spleen cells, and repair injuries of splenic tissue [29]. All these findings suggest the capability of LBP to repair splenic tissue damage in sepsis and ameliorate immunity.

Human leukocyte antigen-DR (HLA-DR) is the major histocompatibility complex II molecules (MHC-II), which is expressed mainly over monocytes, macrophages, dendric cells (DC), and B lymphocytes [30]. In splenic tissue, HLA-DR protein is normally located in splenic macrophages and B lymphocytes and expressed mainly over the cellular membrane. Results of IHC for HLA-DR antigens showed positive expression in the Sham group, manifesting brown staining in a relatively larger area with strong positivity (3+), but without obvious difference between timepoints. The intensity in the positive expression of splenic HLA-DR was reduced in rats in the CLP and LBP groups, with the reduction degree increasing gradually along with time after modeling, while negative expression was noticed in the CLP 18 h group, suggesting the presence of immunosuppression deduced from the gradually decreased expression of HLA-DR in CLP rats along with the prolonged disease. The expression of HLA-DR is indispensable for antigen presentation by monocytes, and the loss of its expression over surface of mononuclear macrophages is the marker for diagnosing sepsis-related immunosuppression and evaluating its prognosis [31, 32]. Upregulation of expression of HLA-DR in monocytes, therefore, may activate immunity against sepsis [33]. It has been revealed by the researchers that LBP may improve the proliferation of splenic cells in rats and upregulate the expression of MHC-II molecules both in macrophages and over the surface of DC cells [12, 33, 34], thereby enhancing systemic immunity. In this research, similarly, the intensity of expression of HLA-DR increased with more obvious findings in the LBP3 group in CLP rats pretreated with LBP in various doses, suggesting the capability of LBP to restore systemic immunity through enhancing HLA-DR expression in the spleen of sepsis rats in a dose-dependent manner.

## 5. Conclusion

In summary, LBP may ameliorate clinical symptoms of rats with cecum ligation perforation, decrease 72-hour mortality, relieve systemic inflammatory reactions, ameliorate splenic injuries, improve cellular immunity in the spleen, and treat sepsis. However, the more profound mechanism with which LBP participates in inflammatory reactions in sepsis and immunity disorder needs further investigations, so as to provide a theoretical basis for pathogenesis and development of sepsis as well as its diagnosis and treatment and offer scientific proofs for development and utilization of LBP applied to critical diseases.

## Figures and Tables

**Figure 1:** Clinical score changes in the Sham, CLP, LBP1, LBP2, and LBP3 groups after CLP and LBP therapy.

**Figure 2:** (a) Neutrophil count, (b) TNF-*α*, (c) IL-10, and (d) lymphocyte count (LYM) changes in the Sham, CLP, LBP1, LBP2, and LBP3 groups after CLP and LBP therapy. ^*∗*^*P* < 0.05, vs. the Sham group; #*P* < 0.05, vs. the CLP group; ▲*P* < 0.05, vs. the LBP1 group; ★*P* < 0.05, vs. the LBP1 group; Δ*P* < 0.05, vs. the 6 h group; ☆*P* < 0.05, vs. the 12 h group, respectively.

**Figure 3:** (a) Spleen index (SI) changes in the Sham, CLP, LBP1, LBP2, and LBP3 groups after CLP and LBP therapy. (b) Quantitative graph.^*∗*^*P* < 0.05, vs. the Sham group; #*P* < 0.05, vs. the CLP group; ▲*P* < 0.05, vs. the LBP1 group; ★*P* < 0.05, vs. the LBP1 group; Δ*P* < 0.05, vs. the 6 h group; ☆*P* < 0.05, vs. the 12 h group, respectively.

**Figure 4:** (a) CD3+ T cells change in the Sham, CLP, LBP1, LBP2, and LBP3 groups after CLP and LBP therapy. (b) Quantitative graph. ^*∗*^*P* < 0.05, vs. the Sham group; #*P* < 0.05, vs. the CLP group; ▲*P* < 0.05, vs. the LBP1 group; ★*P* < 0.05, vs. the LBP1 group; Δ*P* < 0.05, vs. the 6 h group; ☆*P* < 0.05, vs. the 12 h group, respectively.

**Figure 5:** (a) CD4+ T cells change in the Sham, CLP, LBP1, LBP2, and LBP3 groups after CLP and LBP therapy. (b) Quantitative graph. ^*∗*^*P* < 0.05, vs. the Sham group; #*P* < 0.05, vs. the CLP group; ▲*P* < 0.05, vs. the LBP1 group; ★*P* < 0.05, vs. the LBP1 group; Δ*P* < 0.05, vs. the 6 h group; ☆*P* < 0.05, vs. the 12 h group, respectively.

**Figure 6:** (a) CD8+ T cells change in the Sham, CLP, LBP1, LBP2, and LBP3 groups after CLP and LBP therapy. (b) Quantitative graph. ^*∗*^*P* < 0.05, vs. the Sham group; #*P* < 0.05, vs. the CLP group; ▲*P* < 0.05, vs. the LBP1 group; ★*P* < 0.05, vs. the LBP1 group; Δ*P* < 0.05, vs. the 6 h group; ☆*P* < 0.05, vs. the 12 h group, respectively.

**Figure 7:** (a) Immunohistochemical detection of Splenic HLA-DR expression. (b) Splenic HLA-DR integrated optical density (IOD) in rats of various groups. ^*∗*^*P* < 0.05, vs. the Sham group; #*P* < 0.05, vs. the CLP group; ▲*P* < 0.05, vs. the LBP1 group; ★*P* < 0.05, vs. the LBP1 group; Δ*P* < 0.05, vs. the 6 h group; ☆*P* < 0.05, vs. the 12 h group, respectively.

**Table 1:** Summary of groups and subgroups.

Groups	Processing	N
Sham		18
6 h	Saline + Sham	6
12 h	Saline + Sham	6
18 h	Saline + Sham	6

CLP		28
6 h	Saline + CLP	8
12 h	Saline + CLP	8
18 h	Saline + CLP	12

LBP1		18
6 h	LBP 200 mg/kg + CLP	6
12 h	LBP 200 mg/kg + CLP	6
18 h	LBP 200 mg/kg + CLP	6

LBP2		18
6 h	LBP 400 mg/kg + CLP	6
12 h	LBP 400 mg/kg + CLP	6
18 h	LBP 400 mg/kg + CLP	6

LBP3		18
6 h	LBP 800 mg/kg + CLP	6
12 h	LBP 800 mg/kg + CLP	6
18 h	LBP 800 mg/kg + CLP	6

CLP: cecal ligation and puncture.

**Table 2:** Clinical score in rats of various groups.

Groups	Sham	CLP	LBP1	LBP2	LBP3	*F*	*P*
6 h	0.00 ± 0.00	13.63 ± 1.19^*∗*^	11.33 ± 1.86^*∗*^^#^	9.00 ± 2.37^*∗*^^#▲^	7.83 ± 1.60^*∗*^^#▲★^	68.93	≤0.01
12 h	0.00 ± 0.00	15.88 ± 0.99^*∗*^^△^	13.67 ± 1.37^*∗*^^#△^	12.33 ± 1.21^*∗*^^#▲△^	10.05 ± 1.38^*∗*^^#▲★△^	198.13	≤0.01
18 h	0.00 ± 0.00	17.75 ± 0.46^*∗*^^△☆^	16.67 ± 1.51^*∗*^^△☆^	15.17 ± 1.94^*∗*^^#▲△☆^	13.50 ± 1.52^*∗*^^#▲★△^	204.02	≤0.01
*F*	0.00	57.99	16.93	15.83	21.38		
*P*	≤0.01	≤0.01	≤0.01	≤0.01	≤0.01		

^*∗*^ *P* < 0.05, vs. the Sham group; #*P* < 0.05, vs. the CLP group; ▲*P* < 0.05, vs. the LBP1 group; ★*P* < 0.05, vs. the LBP1 group; Δ*P* < 0.05, vs. the 6 h group;☆*P* < 0.05, vs. the 12 h group, respectively.

## Data Availability

The data sets used and/or analyzed during the present study are available from the corresponding author on reasonable request.
